The article "Inhibition of Staphylococcus aureus α-Hemolysin Production Using Nanocurcumin Capped Au@ZnO Nanocomposite" was published in 2022. Journal: Bioinorg Chem Appl.

# Inhibition of *Staphylococcus aureus α*-Hemolysin Production Using Nanocurcumin Capped Au@ZnO Nanocomposite

**DOI:** 10.1155/2022/2663812

**Published:** 2022-05-28

**Authors:** Majid S. Jabir, Taha M. Rashid, Uday M. Nayef, Salim Albukhaty, Faizah A. AlMalki, Jawaher Albaqami, Amal A. AlYamani, Zainab J. Taqi, Ghassan M. Sulaiman

**Affiliations:** ^1^Department of Applied Sciences, University of Technology, Baghdad 10066, Iraq; ^2^Department of Chemistry, College of Science, University of Misan, Maysan 62001, Iraq; ^3^Department of Biology, College of Science, Taif University, P.O. Box 11099, Taif 21944, Saudi Arabia; ^4^Department of Biotechnology, College of Science, Taif University, P.O. Box 11099, Taif 21944, Saudi Arabia

## Abstract

Nanoparticles of gold with zinc oxide (Au@ZnO NPs) were prepared by laser ablation and then capped with curcumin nanoparticles (Cur-Au@ZnO NPs). The synthesized NPs were characterized using different techniques, including transmission electron microscopy (TEM), Fourier-transform infrared spectroscopy (FTIR), UV-visible spectroscopy, and X-ray diffraction. In addition, the ability of NPs as a promising antibacterial agent was tested against *Staphylococcus aureus* through the agar well diffusion method and AO/EtBr staining assay. The results showed that the prepared nanoparticles (Cur-Au@ZnO) served as an antibacterial agent and can destroy the bacterial cells by losing the cell wall integrity and penetrating the cytoplasmic membrane. Moreover, the findings confirmed the role of the formed NPs in attenuation of the adherence and invasion of *S. aureus* to rat embryonic fibroblast (REF) cells. Furthermore, the activity of Cur-Au@ZnO NPs against the *S. aureus α*-hemolysin toxin was evaluated using the western blot technique, using human alveolar epithelial cells (A549), and through histopathology examination in a mouse model. In conclusion, the built Cur-Au@ZnO NPs can be used as a potential antibacterial agent and an inhibitor of *α*-hemolysin toxin secreted by *S. aureus*. These NPs may offer a new strategy in combating pathogen infections and in the future for biomedical and pharmaceutical applications.

## 1. Introduction

*Staphylococcus aureus* (*S. aureus*) is a Gram-positive bacterial strain. It is one of the most well-known and dangerous pathogens in the world's public health concerns. This bacterium can cause osteomyelitis, sepsis syndrome, endocarditis, keratitis, and pneumonia [1]. In addition, *S. aureus* is one of the most common etiological agents of ventilator-associated pneumonia, and it is increasingly recognized as the leading cause of community-acquired pneumonia, affecting otherwise healthy adults and children [2, 3]. The pathogenicity of this bacterial strain is due, in part, to the expression of a large number of virulence genes, including superoxide dismutase, catalase, hyaluronidase, fibrinolysin, hemolysin (alpha, beta, delta, and gamma), superantigens, and epidermolytic toxins [4]. Alpha-Hemolysin (encrypted by the Hla gene), a 33.2 kDa water-soluble monomer secreted by most pathogenic strains of *S. aureus*, targets nearly all mammalian cells by forming stable, amphiphilic transmembrane pores [5, 6]. It is believed to be a critical protein that modulates *aureus* wound healing [7]. In a rat model of *S. aureus*-induced pneumonia, *α*-hemolysin has been shown to destroy the lung's air-blood barrier [8], while *S. aureus* mutant strains lacking *α*-hemolysin are ineffective at causing pneumonia-related mortality. Furthermore, *α*-hemolysin has been demonstrated to be a partial determinant in *S. aureus*-caused ocular infections through various mechanisms [9]. Targeting *α*-hemolysin toward *S. aureus* pneumonia may be a viable alternative approach based on these factors. Although we wait for novel therapeutics or clinical alternatives for the diagnosis and intervention of *S. aureus*, the advancement of treatment interventions is critical.

The article "Inhibition of Staphylococcus aureus α-Hemolysin Production Using Nanocurcumin Capped Au@ZnO Nanocomposite" was published in 2022. Journal: Bioinorg Chem Appl.

Curcumin (1,7-bis (4-hydroxy-3-methoxyphenyl)-1,6-heptadiene-3,5-dione) originating from the *Curcuma longa* rhizomes possesses a variety of biological and pharmacological properties [10]. It has a strong preference for chelating with metal ions and has poor bioavailability and absorption in biological applications due to its incompatibility with water (20 g/mL) [11]. Several distribution methods were established to increase curcumin bioavailability, including nanoparticles, liposomes, microemulsions, vesicles, complexation with phospholipids, and inclusion complexes based on cyclodextrin [12]. Nanomaterials have emerged as a promising potential therapy for overcoming the challenges of treating S. aureus infections due to their capacity to decrease biofilm formation, increase intracellular retention, and improve the antibacterial activity of loaded antimicrobial drugs [13, 14]. Due to their potential to alter the nucleation and growth of nanoparticles, a variety of biomaterials, such as peptides, amino acids, and proteins, have been widely used to manufacture diverse nanomaterials. Because of their bioactive surface, the biomaterial-conjugated nanoparticles were more suited for biological applications [15]. By deliberately realizing the sensors of host cells and bacterial cells, the modified nanomaterials could improve the transmembrane efficiency of everyone's payload compound. Recently, more antimicrobial agents were being formulated into or covalently linked into nanocarriers to improve the pharmacologic activities against sensitive and resistant *S. aureus* and reduce drug side effects [16]. As a result, nanoparticle drug delivery proved to be an excellent tool in overcoming the problems associated with *S. aureus* infection and medicinal plants' bioavailability.

The article "Inhibition of Staphylococcus aureus α-Hemolysin Production Using Nanocurcumin Capped Au@ZnO Nanocomposite" was published in 2022. Journal: Bioinorg Chem Appl.

Nanoparticles can be employed to build structures or nanocomposites that perform a more extensive range of functions than bulk materials. Their surface area-to-volume ratio and nanotechnology proportions with a fantastic size, form, and functions make them unique biological tools [17, 18]. Nanoparticle colloids are modulated with their particular characteristics in the scenario of cell transport, versatility, and numerous fields of study in strength analysis, diagnostic imaging, and chemistry [19–22]. Pulsed laser ablation synthesis is among the best methods compared with wet-chemical syntheses for preparing nanoparticles and applying them to a wide range of applications [23, 24]. The shape and size of the crystal structure can also be examined using the composition of the relevant medium, including laser conditions to boost the mobility of nanocrystal material formation processes. The technique produces a nanometer-scale molecule with a unique property by employing a powerful couple of seconds based on speed in an orientated state [25–27]. Gold nanoparticles (Au NPs) are a more intriguing material that has piqued curiosity due to their apparent benefits. To begin, developers can build Au NPs in various shapes ranging in size from 1 nm to over 100 nm, including round, rod-like, enclosure, and other shapes are examples [28]. A previous study demonstrated that the Au NPs have antibacterial activity against *E. coli*, *Pseudomonas aeruginosa,* and *S. aureus* [29]. The electrical properties of gold nanocomposites are impressive, as are their mechanical properties. Because gold nanocomposites are positively charged, they can be created chemically with a wide range of organic molecules, including medications and genomes, and they can even be synthesized at room temperature [30]. Furthermore, Au NPs are nontoxic and biodegradable, have a distinct surface influence, are ultrathin, include surface plasmon enhancement (SPR) property, and exhibit mesoscopic quantum characteristics [31, 32]. Due to these characteristics, Au NPs are the best choice for several biological applications, including biosensing, clinical diagnostics, and drug development. Other scholars have carried out research extensively about how to make Au NPs and how to use them in biosensing [33]. Zinc oxide nanoparticles are among the relevant metal oxides due to their physicochemical properties [34–37]. These NPs even have excellent UV-blocking, antibiotic, and antibacterial activities. Additionally, ZnO NPs were used successfully in chlorinated cotton fabrics' preparation with fibulas characterization [38]. This study aimed to prepare a new NP tool by applying Au, ZnO, and curcumin using laser ablation and examine their characteristics; additionally, to evaluate the antibacterial activity of the synthesized Cur-Au@ZnO NPs against *S. aureus* pathogenic bacteria using several biochemical and biological techniques; and then study the one possible mechanism by which prepared NPs to kill *S. aureus* through inhibiting the production of bacterial *α*-hemolysin toxin. To our knowledge, the present study is the first to show the antimicrobial properties of the synthesized Cur-Au@ZnO NPs.

The article "Inhibition of Staphylococcus aureus α-Hemolysin Production Using Nanocurcumin Capped Au@ZnO Nanocomposite" was published in 2022. Journal: Bioinorg Chem Appl.

## 2. Materials and Methods

### 2.1. Chemicals and Materials

Chloroauric acid (HAuCl_4_.3H_2_O) was purchased from Sigma, USA. Zinc granulated metal (Zn) at a purity of 99.9% was purchased from VWR International, USA. Muller–Hinton agar and nutrient broth medium were purchased from HiMedia (India). The rat embryonic fibroblast (REF) cell line was kindly gifted from the Iraqi Center for Cancer and Medical Genetics Research (ICCMGR). RPMI-1640 medium was purchased from Gibco (USA). Fetal calf serum, streptomycin, penicillin, acridine orange, ethidium bromide, trypsin-EDTA, and crystal violet stain were purchased from Sigma Chemical Co. (St. Louis, MO, USA). Αlpha-hemolysin and b-tubulin antibodies were purchased from Abcam. Hematoxylin and eosin stains were purchased from Sigma (USA). All other chemicals and reagents were of the analytical grade level.

### 2.2. Microorganism

The antimicrobial efficacy of the prepared NPs was tested against the clinical isolates of *S. aureus*, isolated from the urinary tract and wound infections, respectively. Processing and identification of these isolates were achieved by following the standard biochemical methods at the laboratory. After the transfer of the stock cultures into Mueller–Hinton agar medium, overnight incubation at 37°C, and storage at 4°C were performed.

### 2.3. Nanoparticles Synthesis

#### 2.3.1. Preparation of Au@ZnO Core/Shell Nanoparticles

Zinc oxide (ZnO) and Au@ZnO core/shell were synthesized by pulsed laser ablation of pure granulated zinc metal in deionized water and chloroauric acid, respectively, as described in the method of Rashid and his coworkers [39]. The target was put in the bottom of a glass vessel filled with 3 mL of the used liquid media. A Q-switched Nd-YAG laser (*λ* = 1064 nm) with 7-ns pulse duration was used and adjusted to operate at a 1 Hz repetition rate. The laser pulse energy applied to the target was 800 mJ. The laser beam was focused on the target surface using a lens of a focal length of 120 mm. During this process, the solution was stirred by a mechanical rotator to enhance the growth of the produced nanostructure.

The article "Inhibition of Staphylococcus aureus α-Hemolysin Production Using Nanocurcumin Capped Au@ZnO Nanocomposite" was published in 2022. Journal: Bioinorg Chem Appl.

#### 2.3.2. Preparation of Curcumin-Au@ZnO NPs

Curcumin was mixed with distilled water (dH_2_O) in a ratio of 1 : 10 mg/mL. The extract was formulated using a straightforward procedure, and an ultrasonic water path at 200 Hz, 50°C, was used and then cooled to room temperature. Next, the solvent was centrifuged for 10 min at 4000 rpm. The transmission of the color from dark orange to light yellow indicates the decrease of curcumin particles' size and converts to a nanocurcumin structure. Afterward, the products of the formulation were held in sealed containers.

#### 2.3.3. Characterization of Curcumin-Loaded Au/ZnO NPs

An X-ray diffractometer (XRD-6000, ADX-2700, USA) was employed to characterize the prepared nanoparticles (current = 30 mA; voltage = 40 kV). A Cu K*α* incident beam (*λ* = 1.542 A°) at 2*θ* = 20°–80° was applied to identify the patterns in which the particles were diffracted. Transmission electron microscopy (TEM) was employed using a transmission electron microscope (Zeiss, Germany) operating at 400 kV to examine the nanoparticles' size and shapes. A UV-Vis spectrophotometer (Model-Shimadzu, 1200) was used to characterize Au and ZnO nanoparticle solutions. A double beam UV-Vis was used to show the beams at different conditions in the spectral range (200–1100 nm). An FTIR test was achieved using PerkinElmer Spectrum, USA, at spectral ranges between 4500 and 500 cm^−1^ with an attenuated total reflection mode.

### 2.4. Biological Activities of Cur-Au@ZnO NPs

#### 2.4.1. Antibacterial Efficacy of Cur-Au@ZnO NPs

To test the antibacterial activity of the prepared compound, an agar well diffusion technique was employed against the human pathogen *S. aureus*. Before the culturing process started, 20 mL of Muller–Hinton (M-H) was poured into a Petri dish. The bacteria were captured from the stock culture using a sterile wire loop and streaked onto the surface of the plate. A clean tip was used to drill six mm-diameter channels in the agar plate after the culturing process. The screened nanoparticles were inserted into the channels in the agar plate and then incubated at 37°C for 24 h. The zone of inhibition was examined and measured. The experiments were carried out three times. Additionally, the bacteria were grown on an M-H agar medium at 37°C with 50 mL of nutrient broth to examine the impact of Cur-Au@ZnO NPs on the growth curve. The bacteria were grown until the media had an OD of 0.1 at 600 nm wavelengths, which correlates to 10^8^ (CFU/mL). With gentle agitation, 1 mL of the suspension culture was then applied to the nutrient broth, along with Cur-Au@ZnO NPs, and incubated at 37°C for 12 h. Grade OD was measured using a spectrophotometric method to determine the infection [40, 41].

The article "Inhibition of Staphylococcus aureus α-Hemolysin Production Using Nanocurcumin Capped Au@ZnO Nanocomposite" was published in 2022. Journal: Bioinorg Chem Appl.

#### 2.4.2. Detection of the Bacterial Morphology Changes Using SEM

The use of a scanning microscope observed the morphological changes of the *S. aureus*. The NPs-treated bacteria and the untreated ones were centrifuged at 500 rpm and then washed thrice using PBS at a pH of 7.3. A thin suspended film was formed on a clean silicon chip surface. They were then allowed to air dry at room temperature before patching with 1 mL of a fixing buffer. The slides were cultured at 37°C from one to two hours, after which the solvent was drained using ascending grade methanol, dried in the open air, and then fixed on the SEM stubs, where they were coated with gold for 5 minutes, leaving about 20 nm of gold just on the cells surface. Finally, the gold-coated cells were examined using a scanning electron microscope (Vega III; TESCAN, Czechoslovakia) [42].

#### 2.4.3. Evaluation of Bacterial Cells' Viability

An acridine orange/ethidium bromide (AO/EB) staining technique was used to differentiate the bacterial cell viability of *S. aureus* after treatment with the prepared NPs. The assay was carried out according to the manufacturer protocol. The antibacterial efficacy of the Cur-Au@ZnO NPs against the examined bacterial strain was measured using a fluorescent microscope. 50 *μ*L of the treated samples (bacterial suspension) and untreated one were combined with 50 *μ*L of AO/EB (prepared from 10 g/mL AO/EtBr stock solution) and then left for two minutes. After the staining process, a thin layer of the mixture was transferred to a glass slide, examined under an immunofluorescent microscope (Zeiss Axiovert S100). Acridine orange-stained live cells fluoresce green, whereas ethidium bromide-stained dead cells fluoresce red [43].

#### 2.4.4. Bacterial Adherence Assay

Bacterial strains can infect their hosts through interactions with the receptors on the host cell surface in a process known as adhesion, which is the first step to invasion. In the present study, rat embryonic fibroblast (REF) cells were chosen to examine the built NPs' ability to prevent *S. aureus* infection. The cells were cultured in 12-well tissue culture plates at a density of 1 × 10^5^. After that, they were infected with *S. aureus* at a multiplicity of infection (MOI) ratio of 200 : 1 in the absence and existence of Au, ZnO, Au@ZnO NPs, and Cur-Au@ZnO NPs. The plates were incubated for an hour at 37°C in a 5% CO_2_ incubator and then were washed three times with PBS and fixed in PFA for 15 minutes before being stained with crystal violet dye for 15 minutes.

The article "Inhibition of Staphylococcus aureus α-Hemolysin Production Using Nanocurcumin Capped Au@ZnO Nanocomposite" was published in 2022. Journal: Bioinorg Chem Appl.

#### 2.4.5. Bacterial Invasion Assay

REF cells were again grown in 12-well tissue cultures and then infected with *S. aureus* in the absence and presence of Au, ZnO, Au@ZnO NPs, and Cur-Au@ZnO NPs at a concentration of 100 *µ*g/mL for two hours. The culture medium was discarded, and the REF cells were washed thrice with PBS. A fresh RPMI-1640 medium containing 100 *μ*g/mL gentamicin was added, and the mixture was further incubated for 2 h. The cells were washed three times with PBS and broken down for 20 minutes at 37°C with 0.1% Triton X-100. 10 *μ*L was taken from each well and applied to the nutrient agar, where bacterial cells grew and counted after 20 h. The average bacterium from each well was used to calculate the invasion potential of bacteria. This assay was carried out in triplicate [44].

#### 2.4.6. Immunoblot Analysis for *α*-Hemolysin

*S. aureus* samples were collected after treatment with prepared NPs and electrophoresed in 12% SDS-PAGE after boiling in loading reducing buffer and transferred to polyvinylidene fluoride membrane (PVDF). The membrane was incubated overnight at 4°C in 5% bovine serum albumin in PBS to block free protein-binding sites. Samples were then incubated with rabbit polyclonal antibody to *α*-hemolysin (diluted 1 : 1000), and then they were rinsed three times with PBS. The bound antibody was observed using horseradish peroxidase-conjugated anti-rabbit antiserum at a concentration of 1 : 2000. Amersham ECL Western blotting identification reagents have been used to create the blots by an enhanced chemiluminescence kit and exposed to an X-ray film for visualization.

#### 2.4.7. Live/Dead and Cytotoxicity Assays

In RPMI-1640 medium supplemented with 10% fetal bovine serum, the human lung epithelial cells (A549) were plated in 96-well cells at a density of 1 × 10^1^ cells per well. The cells were cocultured with 100 *µ*L of *S. aureus* suspension with and without Au, ZnO, Au@ZnO NPs, and Cur-Au@ZnO NPs and incubated at 37°C. After 8 h of incubation, the cells were either stained with live/dead (green/red) reagent. A confocal microscope was used to obtain microscopic photographs of stained cells. According to the manufacturer's directions, cell viability was determined by measuring lactate dehydrogenase (LDH) release using the cytotoxicity detection kit. The operation of LDH was calculated using a microplate reader.

#### 2.4.8. Lung Infection Model

Mice were treated following the Animal Research Ethics Committee at the University of Technology. Male mice aged 8 to 10 weeks were anesthetized. *S. aureus* suspension was dropped into the left nare. The infected mice were injected directly with Au, ZnO, Au@ZnO NPs, and Cur-Au@ZnO NPs, for 2 h, after infection, and again at 12-h intervals for a total of 4 doses. The control group was given 100 *μ*L of sterile PBS at about the same time. The mice were also euthanized with anesthesia followed by cervical dislocation before the lungs were placed in 10% formalin. Samples were collected, stained using hematoxylin and eosin, and viewed under a microscope.

The article "Inhibition of Staphylococcus aureus α-Hemolysin Production Using Nanocurcumin Capped Au@ZnO Nanocomposite" was published in 2022. Journal: Bioinorg Chem Appl.

### 2.5. Statistical Analysis

The findings were analyzed using the unpaired *t*-test, which compares studying groups at a significant *p*-value of <0.05.

## 3. Results and Discussion

### 3.1. Characterization of Prepared Nanoparticle

#### 3.1.1. Determination of the Shape and Size

TEM was used to study the characterization of the generated NPs. The images of Au, ZnO, and Au@ZnO NPs prepared by laser ablation in liquid with 1064 nm by energy 800 mJ can be seen in Figure 1. On the one hand, Au NPs are presented as semispherical nanoparticles with an average size of 20 nm that represent Au NPs as a core (Figure 1(a)). On the other hand, ZnO NPs appear like a shell around the surface of Au NPs with an average size of 30 nm (Figure 1(b)). Consequently, the mixing of Au with ZnO leads to an increase in the average size of particles due to the growth of ZnO particles on the surface of Au NPs (Figure 1(c)). Additionally, the curcumin nanoparticles are shown with spherical shapes as nanoclusters (Figure 1(d)), mixed with Au@ZnO NPs (Figure 1(e)). Curcumin is thought to play a critical role in the capping of Au@ZnO NPs to minimize their cytotoxicity and become safer when used in clinical applications (Figure 1(e)).

#### 3.1.2. XRD Analysis

For further determination of the Au@ZnO NPs, the XRD pattern was applied (Figure 2). Drops of the suspensions were placed on Si surfaces and dried by drop-casting. On all samples' XRD patterns, a peak of X-ray photons diffracted from the Si substrate was visible at 2*θ* = 28.6°. Thus, all diffraction peaks for Au@ZnO NPs agree well with the standard JCPDS data cards. Moreover, the diffraction peaks at 2*θ* = 38.2°, 44.6°, and 78.2° correspond to the (111), (200), and (311) planes, respectively, referring to the cubic crystal of the Au NPs and are in excellent agreement with the JCPDS (No. 001-1172). These findings are in agreement with Pan and Wang's data [45]. In addition, the NPs of ZnO were indexed to hexagonal quartzite using JCPDS (No. 01-079-0205), and the typical diffraction peaks were at 2*θ* = 31.8°, 34.5°, 36.3°, 56.7°, 63.0°, 65.1°, and 68.3° corresponding to the (100), (002), (101), (110), (103), (200), and (112) planes. The present data show that the XRD pattern of the zinc oxide nanoparticles with gold (Au@ZnO NPs) is highly similar to that of pure zinc oxide nanoparticles, which means that the gold nanoparticles act as a core and have not affected or disrupted the zinc oxide crystal structure.

The article "Inhibition of Staphylococcus aureus α-Hemolysin Production Using Nanocurcumin Capped Au@ZnO Nanocomposite" was published in 2022. Journal: Bioinorg Chem Appl.

#### 3.1.3. FTIR Spectra of Prepared NPs

The FTIR analysis was carried out to investigate the functional groups of biomolecules involved in capping, viable stabilization, and reduction of prepared NPs. The FTIR spectra of Au, ZnO, and Au@ZnO NPs are shown in Figure 3(a)). The 400–4000 cm^−1^ spectrum was used to measure the absorption spectra. In the FTIR spectra of the samples, several bands can be detected. The large and broad band between 3200 and 3600 cm^−1^ was assigned to the characteristic stretching vibration mode of the water O-H, which changes as the concentration of Au nanoparticles increases. The presence of CO_2_ molecules in the ambient air causes bands around 2076 cm^−1^. The small peak represents carbon dioxide O=C=O stretching at 2356 cm^−1^ and 2333 cm^−1^. Also, the O-H bending vibration mode is assigned to the strong band near 1640 cm^−1^ for Au, ZnO, and Au/ZnO. Besides, the spectra of pure curcumin and Cur-Au@ZnO NPs are presented in Figure 3(b), with the orange line referring to active groups for pure curcumin. The uncoordinated phone's ring vibrations caused the band seen at 1640 cm^−1^. Also, the peaks at 1137 and 3346 cm^−1^ are possibly due to O-H deformation and stretching due to moisture adsorbed on the NPs' surface [46]. When Cur NPs were mixed with Au@ZnO NPs, several peaks disappeared, leaving only four prominent peaks: the broad peak at 670 cm^−1^ showed the predicted Zn-O stretching vibrations and the broad peak at 3455 cm^−1^ was the characteristic O-H stretch [47].

#### 3.1.4. UV-Vis Transmittance Spectrum

The transmittance spectrum wavelengths of the Au, ZnO, Au@ZnO, and Cur-Au@ZnO NP suspensions are depicted in Figure 4(a). It shows the transmittance of Au NPs, ZnO NPs, and Au@ZnO NPs. The peak of pure Au NPs was at 527 nm, and the pure ZnO NPs were at 330 nm. When Au was mixed with ZnO, the transmittance decreased significantly, and a deviation occurred toward the red shift for Au was shifted to 540 nm and the blue shift for ZnO NPs to 323 nm. The present examination results are in line with the previous study by Rojas-Lema et al. [48]. UV transmittance is observed in the Au@ZnO nanocomposites. As a result of the low concentration of Au NPs in the colloidal solution of ZnO NPs, the strongly damped transmittance becomes weak and broad. For Au@ZnO suspension, a prominent peak with a red shift of 540 nm was observed, corresponding to the localized SPR of the partially shaped gold nanoparticles. The UV-visible spectrophotometer for pure curcumin NPs can be seen in Figure 4(b), which shows the peak of the pure curcumin at 364 nm. In contrast, Cur-Au@ZnO NPs show a massive peak for a mixture of nanomaterials, which refers to pure curcumin and its role as a shell capping to cover the surface of ZnO and Au NPs.

The article "Inhibition of Staphylococcus aureus α-Hemolysin Production Using Nanocurcumin Capped Au@ZnO Nanocomposite" was published in 2022. Journal: Bioinorg Chem Appl.

### 3.2. Biological Studies

#### 3.2.1. Antibacterial Activity of Cur-Au@ZnO NPs

*S. aureus* was used to test the antimicrobial properties of Au NPs, ZnO NPs, Cur NPs, Au@ZnO NPs, and Cur-Au@ZnO NPs. Significant inhibition zones were noticed after exposing the organisms to the prepared nanomaterials (Figure 5(a)). The current results indicated the ability of prepared NPs to reduce the bacterial growth rate as indicated in Figure 5(b). The results indicate that the synthesized Cur-Au@ZnO NPs had the highest toxicity against *S. aureus* and inhibited the growth zone by more than 30 mm diameter, particularly after 12 h of exposure, as presented in Figure 5(c). Cur-Au@ZnO NPs were proven to be more effective than other nanoparticles investigated in the present study. Tyagi et al. [49] investigated the cytotoxicity of curcumin at a dosage of 100 *µ*M against 10^6^ CFU/mL *S. aureus* density and reported a 100% killing due to the bacterial membrane damage. Moreover, Bhawana et al. [50] used the wet-milling process to prepare curcumin NPs and investigated their antimicrobial activities against Gram-positive and negative bacterial strains and fungal strains. Their findings demonstrated that the aqueous dispersion of nanocurcumin exhibited significant antimicrobial activity against the chosen bacteria and fungi more than normal curcumin, particularly against *S. aureus*. Additionally, they found that the formed nanocurcumin was more active against bacterial strains than fungal ones. Another study by Sharifi et al. [51] confirmed the effectiveness of nanocurcumin against *E. coli*, *S. aureus, S. pneumonia*, and *Shigella dysenteriae,* which was better than that of the commercial antibiotic amoxicillin. Further, nanocurcumin prevented the formation of biofilm and inhibited the coagulase-negative *Staphylococcus* (CoNS) colonization in nasogastric polyvinyl chloride (PVC) tubes [52]. The antibacterial ability of ZnO nanoparticles has been studied against *B. subtilis*, *S. aureus*, *P. aeruginosa, C. jejuni*, and *E. coli*. Gram-negative bacterial strains have a thin peptidoglycan layer and an outer membrane lipopolysaccharide. An outer membrane acts as a barrier that prevents from entering negatively charged ROS [53]. On the other hand, Gram-positive cell membrane has a less negative charge that allows penetration of negatively charged ROS [54]. The antimicrobial activity of ZnO NPs is related to particle size. It was demonstrated that decreasing the particle size of ZnO NPs results in enhancing antibacterial activity [55]. Another study compared the activity of MgO, TiO_2_, Al_2_O_3_, CuO, CeO_2_, and ZnO nanoparticles against *S. aureus* [56]. Their results demonstrated that ZnO NPs showed significant antibacterial activity. The activity was in a size-dependent manner, and ZnO NPs in different sizes, namely, >1 *μ*m, 8 nm, and 50–70 nm, were used and studied. Their results proved that the small-sized 8 nm ZnO NPs were the best in terms of antibacterial agent. In addition, some studies referred to the toxicity mechanism of metal oxide NPs against bacterial strains related to their size, morphology, and electrostatic attraction [57–59]. Another study done by Jiang et al. [60] reported that the affinity of NPs to aggregate and attach to bacterial surfaces might contribute to NPs' toxicity. Additionally, Aruoja et al. [57] reported that the bactericidal effect of NPs might be specific to the type of metal oxide NPs. It is known that the metal ion NPs have a high affinity for electron-rich molecules such as the genetic material DNA. Moreover, Jose et al. [61] demonstrated that nanoparticles could interact with the isolated DNA molecules and cause a dose-dependent degradation via the generation of single oxygen species. A previous study reported that treatment of bacterial strains with core-shell ZnO and curcumin nanoparticles showed a better bacterial growth inhibition than the commercial antibiotic amoxicillin [62]. Another study demonstrated that the bacterial growth in the presence of curcumin nanoparticles (2–40 nm), attached to the cell wall of the bacterial cell, caused damage to the peptidoglycan layer and then these nanoparticles penetrated inside the cell, which led to disruption of the structure of bacterial cell organelles and killing the bacterial strain through lysis [50]. In a recent study, curcumin was used as an antibacterial agent against *S. aureus* and *E. coli* at concentrations of 200 and 500 *μ*g/mL for 6 h [63]. This study indicated that the conjugation of micro/nanocurcumin particles to ZnO NPs changes the surface charge and hydrodynamic size, thereby enhancing its bioactivity. Curcumin increased the antibacterial activity due to reduced aqueous solubility and exhibited decreased bacterial membrane permeability [64].

The article "Inhibition of Staphylococcus aureus α-Hemolysin Production Using Nanocurcumin Capped Au@ZnO Nanocomposite" was published in 2022. Journal: Bioinorg Chem Appl.

#### 3.2.2. Bacterial Morphology Changes

SEM was used to examine the impact of Au NPs, ZnO NPs, Cur NPs, Au@ZnO NPs, and Cur-Au@ZnO NPs on the formation and structure of *S. aureus* during the study. The photographs revealed variations in the morphology of bacteria cells between the handled and the control samples. Untreated bacterial strain confirmed the cluster-form colonies as illustrated in Figure 6(a). Since *S. aureus* is a Gram-positive bacterium that forms clusters, SEM photos indicate that they would be killed after being treated with Au NPs, ZnO NPs, Cur NPs, Au@ZnO NPs, and Cur-Au@ZnO NPs, as presented in Figures 6(b)–6(f). The prepared NPs under investigation have significant activities against microorganisms. They affected the bacterial strain by colonies damage. This damage was caused by an osmotic imbalance that led to a leak of bacterial cells, resulting in morphological changes, osmotic imbalance, and the cells' structure integrity after being treated with the formed NPs. In comparison with the control group, accumulation and membrane rupture were identified in the *S. aureus* administered with the produced nanoparticles. Many studies examined the bacterial morphological changes after being treated with NPs such as ZnO NPs using SEM and FESEM. The antibacterial activity of ZnO NPs depends on direct contact of ZnO-NPs with the cell walls, resulting in destructing bacterial cell integrity [65, 66]. Another mechanism could be related to the liberation of antimicrobial ions, mainly zinc ions [67], and reactive oxygen species (ROS) formation [68]. Likewise, Bhawana et al. [50] discussed the possible mechanism of action used by nanocurcumin particles to kill bacterial strains, and they reported that the prepared NPs eradicated the bacterial cell wall leading to cell death. Furthermore, for ZnO and Fe_2_O_3_ nanoparticles, the novel antimicrobial agent *α*-Mn_2_O_3_ was prepared by using the hydrothermal technique [69]. *α*-Mn_2_O_3_ NPs showed significant antimicrobial action against *S. aureus ATCC23235*, *B. subtilis ATCC23857*, *E. coli ATCC25922*, *B. pertussis ATCC9797*, and *P. aeruginosa Pao1ATCC15692* bacteria. The morphology changes in bacterial strains after and before treatment of nanorods were examined using SEM analysis. *α*-Mn_2_O_3_ NPs had been indicated huge morphological changes for all tested bacterial strains. In a study by Naskar et al., they synthesized Ni^+2^-doped ZnO NPs. The antibacterial activity of the synthesized nanoparticles was tested against *E. coli ATCC25922*, *A. baumannii ATCC 19606*, *S. aureus ATCC25923*, and *S. epidermidis ATCC 12228* [70]. The morphological changes were studied using the SEM technique. The results showed that the bacterial strains were wrinkling and damaged after exposure to the prepared nanoparticles.

The article "Inhibition of Staphylococcus aureus α-Hemolysin Production Using Nanocurcumin Capped Au@ZnO Nanocomposite" was published in 2022. Journal: Bioinorg Chem Appl.

#### 3.2.3. Evaluation of Bacterial Viability

In this study, the fluorescent microscope and acridine orange-ethidium bromide (AO/EtBr) staining were used to investigate the viability of *S. aureus* after being treated with the prepared NPs (Figure 7). The EtBr contents can only pervade cells' damaged membrane integrity and react with cell nucleic acid. As a result, the viable bacterium will coat green, while the dead cells will stain red [71, 72]. In the current study, *S. aureus* treated with the produced NPs (Au NPs, ZnO NPs, Cur NPs, Au@ZnO NPs, and Cur-Au@ZnO) showed aggressive membrane integrity loss, produced more molecular malformations, and increased in the reddish bacterial numbers. In contrast, untreated cells appeared with an intact and stable structure and bright green color. Khan et al. [73] used Au@ ZnO NPs in *S. aureus* treatment and noticed that the nonviable cells are significantly less at zero-hour incubation, but after 12 h, the percentage of dead cells significantly increased, and cell aggregation was also observed. Generally, the findings revealed that the formed nanoparticles are effective as antibacterial agents and can be applied in biomedical and biological fields. Nagvenkar et al. [74] developed a one-step sonochemical technique to make ZnO-PVA nanoparticles, which were tested against *E. coli* and *S. aureus* using the colony-forming units method and exhibited improved antibacterial activity against both tested bacteria, attributed to its ability to generate ROS, release Zn^+2^ ions, and have antibacterial activity. On the other hand, a study conducted by Alyamani et al. [75] found that ZnO NPs produced by green synthesis using aqueous extracts of *Phlomis* plant had no cytotoxic effect on L929 normal cells but had a significant impact on Gram-positive and Gram-negative bacteria tested. According to Stiefel et al. [76], bacterial viability assays were frequently carried out using a dual staining technique that uses both fluorophores and propidium iodide to detect membrane integrity.

#### 3.2.4. NPs Attenuated the Bacterial Invasion to REF Cells

The REF cells were applied to examine the effect of the synthesized NPs on *S. aureus* attachment and invasion. The cells were handled with 100 *µ*g/mL Au, ZnO, Cur, Au@ZnO, and Cur-Au@ZnO NPs for 1 hour and then infected with *S. aureus* at an MOI (200 : 1) for three hours. As shown in Figure 8, there was a significant decrease in the bacterial infection and attachment to the REF cells when pretreated with Au, ZnO, Cur, Au@ZnO NPs, and Cur-Au@ZnO NPs. Consequently, the invasion of *S. aureus* to the REF cells was dramatically reduced or prevented (Figure 9). Thus, the results of this study indicate that the generated NPs (Au, ZnO, Cur, Au@ZnO NPs, and Cur-Au@ZnO) mediate the adherence and invasion of *S. aureus* strain in REF cells. Likewise, a study by Jihad et al. [44] reported that the pretreated REF cells with graphene oxide nanoparticles capped with polyethylene glycol (PEG) and loaded with *Nigella sativa* (GONPs, GONPs-PEG, and GONPs-PEG-*N. sativa*) at a concentration of 100 *μ*g/mL can delay the invasion of different types of Gram-negative and positive bacterial strains. Taken together, the present study verified that the investigated NPs play a mediation role in the adherence and invasion of *S. aureus* to REF cells.

The article "Inhibition of Staphylococcus aureus α-Hemolysin Production Using Nanocurcumin Capped Au@ZnO Nanocomposite" was published in 2022. Journal: Bioinorg Chem Appl.

#### 3.2.5. Synthesized NPs Block *S. aureus α*-Hemolysin Production

Western blot analysis was used to detect the impact of the formed nanoparticles (Au NPs, ZnO NPs, Cur NPs, Au@ZnO NPs, and Cur-Au@ZnO NPs) on *S. aureus α*-hemolysin production. Alpha-hemolysin is one of the *S. aureus* toxins that target eukaryotic cells, bind to the outer membrane, and form pores causing cell hemolysis and death. Therefore, it is considered the major virulence factor of the pathogen. The results confirmed that the *α*-hemolysin operation in the tested bacteria *S. aureus* was reduced, and the hemolytic behaviors were significantly inhibited, as illustrated in Figure 10. In addition, the investigated nanoparticles were able to abolish or block the *S. aureus α*-hemolysin formation. A previous study [77] investigated the effect of biosynthesized silver nanoparticles (SNPs) on the mRNA expression level, and they reported that the formed SNPs exhibited a significant reduction in the production of this toxin even at doses less than the minimum inhibitory concentration (MIC) value of SNPs. These results are consistent with the current study findings. A preprint has previously been published (DOI: https://doi.org/10.21203/rs.3.rs-516417/v1), and it revealed that Cur-Au@ZnO NPs protect from bacterial infection through inhibiting production of *α*-hemolysin [78].

#### 3.2.6. Prepared NPs Protect Alveolar Epithelial Cells from *S. aureus* Injury

The ability of prepared NPs to prevent *α*-hemolysin-mediated alveolar epithelial cell injury was investigated using the A549 cell line and coculture method. The cell death was evident by an increase in the number of orange-red fluorescent dead cells and a transformation in the cellular morphology of the live cells after coculturing with *S. aureus* (Figure 11). Supplementing the coculture system with Au NPs, ZnO NPs, Cur NPs, Au@ZnO NPs, and Cur-Au@ZnO NPs protected the cells from damage by *S. aureus*. Additionally, the efficacy of the built NPs was further examined using LDH release method, and the results confirmed that the percentage of LDH generated was decreased when Au NPs, ZnO NPs, Cur NPs, Au@ZnO NPs, and Cur-Au@ZnO NPs were supplemented to the coculture of A549 cells and *S. aureus* (Figure 12).

The article "Inhibition of Staphylococcus aureus α-Hemolysin Production Using Nanocurcumin Capped Au@ZnO Nanocomposite" was published in 2022. Journal: Bioinorg Chem Appl.

#### 3.2.7. Cur-Au@ZnO NPs Recover Lung Injury Caused by *S. aureus*

The potential effect of the Cur-Au@ZnO NPs against *S. aureus* was further examined *in vivo* using mice models. The collected data showed that the lung tissue of the infected mice with *S. aureus* and then given PBS were kermesinus and had a firm texture. Additionally, the mice demonstrated significant alveolar disruption and massive numbers of inflammatory cells (Figure 13(b)). In contrast, mice treated with the synthesized NPs (Au, ZnO, Cur, Au@ZnO, and Cur-Au@ZnO) represented open and contained alveoli, with no significant areas of inflammation, although occasionally small areas of congestion as illustrated in Figure 13(c)–13(g). A recent investigation by Wang et al. [79] showed that the formed nanocomposite films, AGO, represented antibacterial activity against *E. coli* and *S. aureus* at a low dose and improved wound healing. The *in vivo* experiment findings demonstrated that the prepared NPs in the current study could stimulate the immune response to produce various types of white blood cells (WBCs) that produce synergistic antibacterial effects and accelerated wound healing.

## 4. Conclusion

To our knowledge, the present study is the first to show the antimicrobial properties of the synthesized Cur-Au@ZnO NPs. Gold with zinc oxide nanoparticles (Au@ZnO NPs) was prepared by laser ablation and then capped with curcumin nanoparticles. The antimicrobial effect of nanocurcumin-Au@ZnO nanocomposite against *S. aureus* was examined. The findings showed that the bacterial strain could be penetrated by the tested NPs, resulting in bacterial strain destruction. In addition, the obtained results demonstrated that the Cur-Au@ZnO NPs are a selective inhibitor of *S. aureus*-secreted *α*-hemolysin. Consequently, the prepared NPs mediated the blocking of *α*-hemolysin activity, which could be a novel way to prevent pathogens' infections. In the future, the formed Cur-Au@ZnO NPs could be applied in clinical trials and biomedical applications as an antimicrobial new agent.

## Figures and Tables

**Figure 1:** TEM images illustrate the size and shape of the synthesized nanoparticles. (a) Au NPs, (b) ZnO NPs, (c) Au@ZnO NPs, (d) Cur NPs, and (e) Cur-Au@ZnO NPs.

**Figure 2:** XRD patterns of Au@ZnO NPs.

**Figure 3:** FTIR spectrum of the prepared nanoparticles. (a) Au NPs, ZnO NPs, and Au@ZnO NPs. (b) Cur NPs and Cur-Au@ZnO NPs.

The article "Inhibition of Staphylococcus aureus α-Hemolysin Production Using Nanocurcumin Capped Au@ZnO Nanocomposite" was published in 2022. Journal: Bioinorg Chem Appl.

**Figure 4:** UV-Vis spectrum. (a) Au NPs, ZnO NPs, and Au@ZnO NPs. (b) Cur NPs and Cur-Au@ZnO NPs.

**Figure 5:** Antibacterial activity of prepared NPs against *S. aureus*. (a) Zone of inhibition: (A) control untreated bacterial strain. The bacterial strains were treated with NPs as follows: (B) ZnO NPs, (C) Cur NPs, (D) Au NPs, (E) Au@ZnO NPs, and (F) Cur-Au@ZnO NPs. (b) A chart diagram for the same results, illustrating the *S. aureus* growth rate for the same treated groups. The data are shown as the mean ± SD. ^*∗∗*^*p* < 0.01, ^*∗∗∗*^*p* < 0.001, and ^*∗∗∗∗*^*p* < 0.0001.

**Figure 6:** SEM images visualized the NPs-treated *S. aureus*. Treated bacterial strains are indicated in red arrows, showing bacterial colonies damage. (a) Control untreated. The *S. aureus* bacteria were treated with NPs as follows: (b) ZnO NPs, (c) Cur NPs, (d) Au NPs, (e) Au@ZnO NPs, and (f) Cur-Au@ZnO NPs.

**Figure 7:** Fluorescence microscopic images of the green and red fluorescence-stained *S. aureus*. (a) Control untreated bacterial strain. The bacterial strain was treated with NPs as follows: (b) ZnO NPs, (c) Cur NPs, (d) Au NPs, (e) Au@ZnO NPs, and (f) Cur-Au@ZnO NPs. Magnification power 40x.

**Figure 8:** The prepared NPs decrease the interaction of *S. aureus* with the REF cells. (A) REF, infected with *S. aureus*. The REF cells were pretreated with NPs and then infected with *S. aureus.* The treatment groups were as follows: (B) with ZnO NPs, (C) with Cur NPs, (D) with Au NPs, (E) with Au@ZnO NPs, and (F) with Cur-Au@ZnO NPs. The values are shown as the mean ± SD. ^*∗∗∗*^*p* < 0.001, ^*∗∗∗∗*^*p* < 0.0001.

**Figure 9:** The prepared NPs inhibit the invasion of *S. aureus* to REF cells. (a) Control REF cells. (b) REF, infected with *S. aureus*. The REF cells were pretreated with NPs and then infected with *S. aureus.* The treatment groups were as follows: (c) with ZnO NPs, (d) with Cur-NPs, (e) with Au NPs, (f) with Au@ZnO NPs, and (g) with Cur-Au@ZnO NPs. Magnification power 400x.

**Figure 10:** Western blot analysis of *α*-hemolysin showed that the synthesized NPs reduced the production of *α*-hemolysin. (A) Control group. The other groups of *S. aureus* were treated with NPs as follows: (B) ZnO NPs, (C) Cur NPs, (D) Au NPs, (E) Au@ZnO NPs, and (F) Cur-Au@ZnO NPs. The graph represented densitometry quantification of the *α*-hemolysin/b-tubulin ratio, as indicated.

**Figure 11:** Cur-Au@ZnO NPs blocked *S. aureus*-mediated lung cell injury. (a) Control A549 cells. (b) A549 cells infected with *S. aureus*. The other groups of A549 cell line were treated with NPs as follows: (c) ZnO NPs, (d) Cur-NPs, (e) Au NPs, (f) Au@ZnO NPs, and (g) Cur-Au@ZnO NPs and then infected with *S. aureus*. Scale bar was 10 *µ*m.

The article "Inhibition of Staphylococcus aureus α-Hemolysin Production Using Nanocurcumin Capped Au@ZnO Nanocomposite" was published in 2022. Journal: Bioinorg Chem Appl.

**Figure 12:** Cur-Au@ZnO NPs reduce LDH release in A549 cells. (A) A549 cells infected with *S. aureus*. Each group of A549 cells was exposed to different NPs being before infected with *S. aureus.* The pretreatments were as follows: (B) with ZnO NPs, (C) with Cur-NPs, (D) with Au NPs, (E) with Au@ZnO NPs, and (F) with Cur-Au@ZnO NPs. The data are shown as the mean ± SD. ^*∗∗*^*p* < 0.01, ^*∗∗∗*^*p* < 0.001.

**Figure 13:** Histopathological changes in lung sections. (a) Control mice lung. (b) Mice were infected with *S. aureus* via the intranasal route and were given the PBS. The other groups of mice were infected with *S. aureus* via the intranasal route and then treated as follows: (c) with ZnO NPs, (d) with Cur NPs, (e) with Au NPs, (f) with Au@ZnO NPs, and (g) with Cur-Au@ZnO NPs. Mice lungs were stained by using hematoxylin and eosin stain. Magnification power 40x.

## Data Availability

The data used to support the findings of this study are included in the article.
